# Effect of Compound Polyethylene Glycol Electrolyte Powder on the Quality of Gastrobowel Preparation before Enteroscopy Intervention

This article has been retracted.

**DOI:** 10.1155/2022/9895499

**Published:** 2022-08-31

**Authors:** Yongxin Yuan, Yuqin Li, Yafeng Zhang, Jing Jiang, Yi He, Yimei Liao, Wenchun Yao

**Affiliations:** ^1^Department of Anorectal, Suining Central Hospital, Suining, Sichuan 629000, China; ^2^Department of Nuclear Medicine, Suining Central Hospital, Suining, Sichuan 629000, China

## Abstract

**Objective:**

To study the effect of compound polyethylene glycol electrolyte powder (PGEP) on the quality of gastrobowel preparation before enteroscopy intervention.

**Methods:**

From March 2021 to January 2022, among the patients who needed enteroscopy in our hospital, 280 patients who volunteered for this study were randomly selected as the research objects. All the subjects were randomly divided into the control group (140 cases) and the observation group (140 cases). Both groups received routine treatment before enteroscopy intervention. On this basis, patients in the control group were given 9 g of senna every day before operation, and 250 ml of 20% mannitol and 2500 ml of water were taken orally from 9:00 am to 11:00 am on the day of examination. Patients in the observation group took PGEP orally from 9:00 am to 11:00 am. The effective rate of bowel cleaning, the frequency of defecation and duration of diarrhea, the levels of blood electrolyte indexes such as Na^+^, K^+^, and Cl^−^ before and after the intervention, and the incidence of adverse reactions were compared between the two groups.

**Results:**

The effective rate of bowel cleaning in the observation group was significantly higher than that in the control group (*P* < 0.05). The frequency of defecation and duration of diarrhea in the observation group were significantly lower than those in the control group (*P* < 0.05). Compared with the control group, the levels of blood electrolyte indexes in the observation group after the intervention were not statistically significant (*P* > 0.05). The incidence of adverse reactions in the observation group was significantly lower than that in the control group (*P* < 0.05).

**Conclusion:**

Using PGEP for gastrobowel preparation before enteroscopy intervention can achieve high bowel cleaning efficiency, short bowel preparation time, and low incidence of adverse reactions, which does not affect the water-electrolyte balance of patients, and the psychological state of patients before enteroscopy intervention is more stable. This program is worthy of clinical promotion.

## 1. Introduction

Enteroscopy is the most commonly used and accurate method to observe the colonic mucosa, and it is the gold standard for the diagnosis of many colorectal diseases [1]. In enteroscopy, the electronic camera located at the front end can accurately transmit the patient's bowel mucosa to the electronic computer. The examining doctor can observe the smallest changes of the mucosa at the enteroscopy, but the clarity of the image mainly depends on the bowel cleanliness of the patient [2]. The study shows that good bowel cleanliness can greatly improve the inspection effect of enteroscopy [3]. Traditional bowel preparation is mainly based on oral senna 3 days before operation and 20% mannitol catharsis before operation. If necessary, cleaning enema is added. The bowel cleaning effect is not good, and the preparation time is long [4]. Traditional bowel preparation requires a long time for patients' preoperative diet control, and high-pressure enema may cause adverse reactions such as bowel edema and ascites. Patients are prone to anxiety and irritability and other bad emotions, which increases the difficulty of nursing work and reduces the accuracy of enteroscopy [5]. Therefore, it has been a hot topic in clinical research to find a more effective and safe bowel preparation plan. The ideal bowel preparation plan should completely reduce bowel contents, reduce bowel bacteria to a minimum, make patients comfortable and actively cooperate, and not interfere with patients' internal homeostasis [6]. Oral electrolyte method is the latest bowel preparation method. Its operation method omits the steps of oral senna and enema, and the preoperative diet control time is relatively short, which is simple and easy to implement, and the incidence of adverse reactions is lower, and patients' compliance is higher, which is very helpful for the development of nursing work [7]. At present, the electrolyte powder is mainly compound polyethylene glycol electrolyte powder (PGEP), which is an impermeable oral laxative [8]. At present, it has been widely used in bowel preparation before colorectal surgery, enteroscopy, and gynecological pelvic tumor surgery. It can not only reduce the pain of bowel preparation for patients but also ensure good bowel cleanliness, which is convenient for operation and has high safety [9, 10]. We carried out further research on gastrobowel preparation before enteroscopy intervention, and the report is as follows.

## 2. Data and Methods

### 2.1. General Information

From March 2021 to January 2022, among the patients who needed enteroscopy in our hospital, 280 patients who volunteered for this study were randomly selected as the research objects. The inclusion criteria were as follows: ① age ≥ 18 years old; ② they had abdominal pain, diarrhea, melena, bloody stool, change of stool habits, abdominal mass and other clinical manifestations, and suspected colon, rectum, and terminal ileum lesions, so they needed enteroscopy; ③ according to the evaluation of the investigator, the subjects met the study requirements, were able to communicate with the investigator about the preoperative bowel preparation method, volunteered to participate in the study, and signed the informed consent form. Exclusion criteria were as follows: ① complicated with severe gastrointestinal diseases such as obvious bowel obstruction, bowel inflammation, stenosis, severe constipation, and other diseases; ② complicated with severe immune system diseases or advanced malignant tumor; ③ complicated with severe cardiovascular and cerebrovascular diseases and liver and kidney diseases; ④ there is a history of allergy or intolerance to compound polyethylene glycol; ⑤ emergency surgery patients; and ⑥ pregnant and lactating women. All the subjects were randomly divided into the control group (140 cases) and the observation group (140 cases). There were 88 males and 52 females in the control group, with an average age of (48.10 ± 3.24) years, and 89 males and 51 females in the observation group, with an average age of (48.42 ± 3.81) years. There was no significant difference in gender, age, and other general information between the two groups (*P* > 0.05), which could be used for experimental comparison.

### 2.2. Methods

Both the observation group and the control group were given semi-liquid diet on the 3rd day before operation and full-liquid diet on the 1st day and 2nd day before operation. Patients in the control group were given 9 g of senna every day before operation, and 250 ml of 20% mannitol and 2500 ml of water were taken orally from 9:00 am to 11:00 am on the day of examination. If necessary, 0.90% saline was added for enema. The patients in the observation group took PGEP (produced by Jiangxi Hengkang Pharmaceutical Co., Ltd., Guoyao Zhunzi h20020031) orally from 09:00 to 11:00 a.m. on the day of examination. 3000 ml solution was prepared according to the instructions, 600-1000 ml solution was taken for the first time, and then 250 ml solution was taken once every 10-15 minutes, until the water sample was discharged to clear the stool. Closely observe the patients to prevent serious complications. Both groups of patients need to move around as much as possible after taking the medicine and are not allowed to stay in bed or sit for a long time.

### 2.3. Observation Index

① Compare the bowel cleaning efficiency of the two groups. ② The frequency of defecation and duration of diarrhea were compared between the two groups. ③ The venous blood of the subjects was drawn, and the levels of blood electrolyte indexes such as Na^+^, K^+^, and Cl^−^ were compared before and after intervention. ④ The incidence of adverse reactions such as abdominal distension, abdominal pain, nausea and vomiting, and fatigue during bowel preparation were compared between the two groups.

### 2.4. Bowel Cleaning Standards

Cleanliness of bowel tract: grade I—no feces or residues are found in the bowel tract, no retention of feces and water, clear bowel fluid, smooth operation, and unaffected observation; grade II—there is no fecal residue in the bowel cavity, but there is less dirty fecal water, so the operation is smooth and the observation is basically clear; and grade III—there are fecal residues or fecal lumps in the bowel cavity, so the operation is not smooth and the operation is greatly affected.

(1) $$\begin{array}{c} \text{The effective rate of bowel cleaning}=\frac{\text{grade I}+\text{grade II}}{\text{total number}}\times 100\%. \end{array}$$

Frequency of defecation: the total number of defecations of the patient after medication until bowel preparation before enteroscopy intervention.

Duration of diarrhea: the number of days that diarrhea lasted for the patient after medication until bowel preparation before enteroscopy intervention.

### 2.5. Statistical Method

SPSS 22.0 professional statistical software was used to analyze all statistical data. The measured data were expressed as mean ± standard deviation, *t*-test was used for comparison, all count data were expressed as rate (*n*, %), and *χ*^2^ test was used for comparison. *P* < 0.05 was evaluated as significant difference.

## 3. Results

### 3.1. Comparison of Bowel Cleaning Efficiency between Two Groups of Patients

The effective rate of bowel cleaning in the observation group was 92.86%, and the effective rate of bowel cleaning in the control group was 76.43%. The effective rate of bowel cleaning in the observation group was significantly higher than that in the control group (*P* < 0.05) (see Table 1 for details).

### 3.2. Comparison of Diarrhea Duration and Defecation Times between the Two Groups

The frequency of defecation and duration of diarrhea in the observation group were significantly lower than those in the control group (*P* < 0.05) (see Table 2 for details).

### 3.3. Comparison of Blood Electrolyte Indexes between the Two Groups before and after Intervention

Before and after the intervention, there was no significant difference in the levels of Na^+^, K^+^, and Cl^−^ and other blood electrolyte indexes between the two groups (*P* > 0.05). Compared with the control group, the levels of blood electrolyte indexes in the observation group after the intervention were not statistically significant (*P* > 0.05) (see Table 3 for details).

### 3.4. Comparison of the Incidence of Adverse Reactions between the Two Groups

The incidence of adverse reactions in the observation group was 17.14%, and the incidence of adverse reactions in the control group was 29.28%. The incidence of adverse reactions in the observation group was significantly lower than that in the control group (*P* < 0.05) (see Table 4 for details).

## 4. Discussion

It is a clinical consensus that effective bowel preparation should be carried out for patients before enteroscopy. The standard of bowel preparation is that the colon is empty, clean, collapsed, and sterile, and there are few adverse reactions, which have little impact on the patient's psychological state [11]. Traditional bowel preparation methods mainly include oral catharsis and clean enema, that is, the patients' diet is controlled 3 days before operation, and oral laxatives and artificial enema are required. Studies have shown that the traditional bowel preparation methods have low bowel cleaning efficiency, and long-term dietary control tends to aggravate adverse reactions such as negative nitrogen balance, metabolic disorder, and decreased subjective tolerance [12]. At the same time, the operation of bowel preparation is difficult, causing serious irritation to gastrobowel tract. Mannitol used for bowel preparation may produce a large amount of explosive gases (methane and hydrogen) after being decomposed by bacteria, which may lead to abdominal pain, abdominal distension, bowel obstruction, bowel bleeding, and other complications [13]. At the same time, studies have confirmed that repeated enema may increase the pain of patients, and patients may have negative emotions such as anxiety and depression, so it is difficult to carry out clinical practice [14]. In recent years, the new bowel preparation method is mainly oral electrolyte method. Its main action principle is that a large amount of electrolyte-containing liquid enters the bowel tract in a short time and can stay in the bowel canal by its own gravity, directly stimulating the bowel wall mucosa, enhancing its peristalsis, softening feces, and promoting defecation [15, 16]. At present, this method has been widely used in preoperative preparation for colorectal tumor resection, preoperative preparation for gynecological diseases, and preoperative preparation for enteroscopy, and its safety and effectiveness have been confirmed by a large number of studies at home and abroad.

PGEP is the most commonly used electrolyte powder in clinic, which is composed of polyethylene glycol, sodium bicarbonate, sodium sulfate, potassium chloride, and sodium chloride [17]. Pharmacological studies have shown that its main component polyethylene glycol can stably combine with water molecules in bowel contents through hydrogen bonds without being absorbed by the colon, thereby making manure water become isotonic liquid, thus balancing the osmotic pressure inside and outside the bowel mucosa [18]. PGEP can reduce the absorption of bowel mucosa, having the characteristics of non-absorption and non-secretion [19, 20]. Bowel bacteria have a weak decomposition effect on it, with high safety, and the incidence of abdominal pain, abdominal distension, bowel obstruction, and other adverse reactions is low [21, 22]. At the same time, its action time is short, and dehydration and water-electrolyte disorder will not be caused by excessive extravasation of liquid [23]. PGEP is used for bowel preparation before enteroscopy, colorectal cancer resection, and gynecological surgery, which not only saves long-term diet control but also has the characteristics of simplicity and ease of use. After taking the medicine, the bowel cleanliness is high, which will not increase the pain of patients. The patient's compliance is high and the psychological state is good [24, 25]. The results of this study showed that the effective rate of bowel cleaning in the observation group was significantly higher than that in the control group (*P* < 0.05), and the frequency of defecation and duration of diarrhea in the observation group were significantly lower than those in the control group (*P* < 0.05), which suggested that PGEP had a rapid and effective role in bowel preparation. The incidence of adverse reactions in the observation group was significantly lower than that in the control group (*P* < 0.05), and the levels of blood electrolytes in the two groups were not significantly different from those before the intervention (*P* > 0.05). This reflects the non-secretion and non-absorption characteristics of PGEP. PGEP is isotonic in nature, with less fluid exchange and lower incidence of water-electrolyte disturbance, which had less impact on the patient's internal homeostasis and had high safety.

To sum up, using PGEP for gastrobowel preparation before enteroscopy intervention can achieve high bowel cleaning efficiency, short bowel preparation time, and low incidence of adverse reactions, which does not affect the water-electrolyte balance of patients, and the psychological state of patients before enteroscopy intervention is more stable. This program is worthy of clinical promotion. This study has some limitations. It is not only a single-center study with a small sample size but also lacks objective evaluation criteria for adverse reactions. We need to further improve this research to provide evidence for clinical practice.

## Figures and Tables

**Table 1:** Comparison of bowel cleaning efficiency between two groups of patients (*n* (%)).

Group	Grade I	Grade II	Grade III	Total effective rate
Control group (*n* = 140)	45 (32.14%)	62 (44.29%)	33 (23.57%)	107 (76.43%)
Observation group (*n* = 140)	61 (43.57%)	69 (49.29%)	10 (7.14%)	130 (92.86%)
*χ* ^2^	—			14.53
*P*	—			0.00

**Table 2:** Comparison of bowel preparation time between two groups ($\bar{x}\pm s$).

Group	Frequency of defecation (times)	Duration of diarrhea (h)
Control group (*n* = 140)	6.19 ± 1.22	6.36 ± 0.82
Observation group (*n* = 140)	4.41 ± 1.05	3.81 ± 0.63
*t*	8.92	18.47
*P*	0.00	0.00

**Table 3:** Comparison of blood electrolyte indexes between the two groups before and after intervention ($\bar{x}\pm s$).

Group	Na^+^ (mmol/L)		K^+^ (mmol/L)		Cl^−^ (mmol/L)	
	Before intervention	After intervention	Before intervention	After intervention	Before intervention	After intervention
Control group (*n* = 140)	138.44 ± 3.98	137.88 ± 2.70	4.31 ± 0.53	3.89 ± 0.43^①^	104.36 ± 2.59	102.67 ± 2.24^①^
Observation group (*n* = 140)	138.29 ± 3.33	137.14 ± 2.52^①^	4.39 ± 0.60	3.77 ± 0.54^①^	104.78 ± 2.66	101.89 ± 2.11^①^
*t*	2.23	1.68	0.80	1.31	1.06	2.06
*P*	>0.05	>0.05	>0.05	>0.05	>0.05	>0.05

*Note.* Compared with before intervention, ^①^*P* < 0.05.

**Table 4:** Comparison of the incidence of adverse reactions between the two groups (*n* (%)).

Group	Abdominal distention	Abdominal pain	Nausea and vomiting	Fatigue	Total number of adverse reactions
Control group (*n* = 140)	15 (10.71%)	10 (7.14%)	7 (5.00%)	9 (6.43%)	41 (29.28%)
Observation group (*n* = 140)	9 (6.43%)	8 (5.71%)	3 (2.14%)	4 (2.86%)	24 (17.14%)
*P*	0.01				
*χ* ^2^	5.79				

## Data Availability

The data used and/or analyzed during the current study are available from the corresponding author upon request.
